The article "The different effector function capabilities of the seven equine IgG subclasses have implications for vaccine strategies" was published in 2008. Journal: Mol Immunol.

# The different effector function capabilities of the seven equine IgG subclasses have implications for vaccine strategies

**DOI:** 10.1016/j.molimm.2007.06.158

**Published:** 2008-02

**Authors:** Melanie J. Lewis, Bettina Wagner, Jenny M. Woof

**Affiliations:** a Division of Pathology and Neuroscience, University of Dundee Medical School, Ninewells Hospital, Dundee DD1 9SY, UK; b Department of Population Medicine and Diagnostic Sciences, College of Veterinary Medicine, Cornell University, Ithaca, NY 14853, USA

**Keywords:** reqIgG, recombinant equine IgG, EHV-1, equine herpes virus-1, NIP, 3-nitro-4-hydroxy-5-iodophenylacetate, PBS-T, PBS-Tween, FcγR, receptor specific for the Fc region of IgG, PBL, peripheral blood leukocyte, Horse, IgG, Recombinant antibodies, Complement, Respiratory burst, Protein A

## Abstract

Recombinant versions of the seven equine IgG subclasses were expressed in CHO cells. All assembled into intact immunoglobulins stabilised by disulphide bridges, although, reminiscent of human IgG4, a small proportion of equine IgG4 and IgG7 were held together by non-covalent bonds alone. All seven IgGs were *N*-glycosylated. In addition IgG3 appeared to be *O*-glycosylated and could bind the lectin jacalin. Staphylococcal protein A displayed weak binding for the equine IgGs in the order: IgG1 > IgG3 > IgG4 > IgG7 > IgG2 = IgG5 > IgG6. Streptococcal protein G bound strongly to IgG1, IgG4 and IgG7, moderately to IgG3, weakly to IgG2 and IgG6, and not at all to IgG5. Analysis of antibody effector functions revealed that IgG1, IgG3, IgG4, IgG5 and IgG7, but not IgG2 and IgG6, were able to elicit a strong respiratory burst from equine peripheral blood leukocytes, predicting that the former five IgG subclasses are able to interact with Fc receptors on effector cells. IgG1, IgG3, IgG4 and IgG7, but not IgG2, IgG5 and IgG6, were able to bind complement C1q and activate complement via the classical pathway. The differential effector function capabilities of the subclasses suggest that, for maximum efficacy, equine vaccine strategies should seek to elicit antibody responses of the IgG1, IgG3, IgG4, and IgG7 subclasses.

## 1 Introduction

Only recently has the full complement of horse Ig heavy (H) chain constant region genes (one δ, one μ, seven γ, one α and one ɛ) been described (Wagner et al., 2004). The horse has the highest number of IgG constant region (γ or *IGHG*) genes of any mammalian species examined to date and all the seven IgG subclasses they encode appear to be expressed *in vivo* (Wagner et al., 2004). Early studies described five equine IgG subclasses named IgGa, IgGb, IgGc, IgG(T), and IgG(B) or ‘aggregating immunoglobulin’. Following identification of the seven horse heavy chain constant region genes, the IgG subclasses have been reassigned as IgG1 to IgG7 (Wagner, 2006). Of the originally described IgG subclasses, IgGa corresponds to IgG1, IgGb to IgG4 and IgG7, IgGc to IgG6, and IgG(T) to both IgG3 and IgG5 (Wagner et al., 2002, 2004).

IgG is the predominant antibody class in equine serum and colostrum (Sheoran et al., 2000) and is present at the mucosal surfaces, where it is the most abundant isotype in the equine urinary tract, lower respiratory tract and lung (Butler, 1998). In equine serum, IgGb (IgG4 and IgG7) is the most prevalent isotype followed by IgG(T) (IgG3 and IgG5), IgGa (IgG1) and IgGc (IgG6). In colostrum, IgGb is predominant, followed by IgGa and IgG(T), while IgGc is barely detectable. In nasal wash samples from adult horses only the IgGa and IgGb subclasses have been detected (Sheoran et al., 2000). Systemic and/or mucosal IgG antibody responses are known to play an important role in protection against several equine pathogens including equine influenza virus (Nelson et al., 1998; Breathnach et al., 2006) and *Streptococcus equi* (Galan and Timoney, 1985; Galan et al., 1986; Sheoran et al., 1997), and may limit the severity and spread of equine herpes virus (EHV)-1 (Kydd et al., 2006).

Although a role for equine IgG antibodies in protection against disease has long been recognised, the structures and functions of the individual IgG subclasses are not well characterised. Identification and cloning of the full complement of IgG H chain genes has provided a fresh resource for the study of equine IgG proteins. Here, we describe the first expression of recombinant versions of all seven equine IgG subclasses and present an analysis of their individual physical and biological properties.

## 2 Materials and methods

### 2.1 Construction of equine γ H chain expression vectors

The mouse V_H_ gene specific for NIP was subcloned as a HindIII-BamHI fragment from a previously described human IgA1 expression vector (Morton et al., 1993) into pcDNA3.1/Hygro (+) (Invitrogen, Paisley, UK) to produce pcDNA3.1Vnip. Isolation of genomic DNA for equine *IGHG3, IGHG4* and *IGHG7*, and cDNA for equine *IGHG1*, *IGHG2*, *IGHG5* and *IGHG6* has been previously described (Wagner et al., 2002, 2004). For construction of the equine IgG3 H chain vector, a 2.5 kb BamHI fragment containing the *IGHG3* gene along with 630 bp of 5′ UTR and 577 bp of 3′ UTR was placed downstream of the mouse V_H_ gene in pcDNA3.1Vnip. To construct mammalian expression vectors for the remaining six horse IgGs, each γ constant region was amplified by PCR and placed downstream of the 630 bp horse *IGHG3* 5′ UTR (also amplified by PCR) within the cloning vector pBluescript II (Stratagene, Amsterdam, The Netherlands). For each subclass, the 5′ UTR and γ constant region cassette was then subcloned into pcDNA3.1VNip downstream of the mouse V_H_ gene.

### 2.2 Expression of reqIgGs in CHO-K1 cells

CHO-K1 cells, which had previously been stably transfected with the mouse λ L chain specific for NIP, were transfected with one of the γ1–γ7 H chain expression vectors, as previously described (Morton et al., 1993). Supernatant from individual resistant CHO clones was screened for Ig production by antigen-capture ELISA as previously described (Morton et al., 1993) except that the detection antibodies used were either rabbit anti-mouse λ L chain–HRP conjugate (0.25 μg/ml in PBS-0.5% Tween [PBS-T]) or goat anti-horse IgG Fc-HRP conjugate (0.4 μg/ml in PBS-T) (both Rockland, Gilbertsville, PA, USA).

### 2.3 Purification and analysis of reqIgGs

ReqIgGs were purified using NIP-affinity chromatography as previously described (Morton et al., 1993), then subjected to gel filtration on a Superose6 column using an ÄKTA FPLC system (GE Healthcare, Little Chalfont, UK). Only fractions corresponding to intact antibody (H_2_L_2_) were pooled for further analysis. The antibodies were analysed by SDS-PAGE and Western blotting on 8.4% acrylamide gels under reducing and non-reducing conditions. Gels were stained with Coomassie brilliant blue and Western blots were probed with HRP-conjugated rabbit anti-mouse λ L chain (0.2 μg/ml) or anti-horse IgG antibodies. Horse serum IgG (Sigma–Aldrich, Poole, UK) and recombinant human IgG1 (Pleass et al., 1999) were used as controls.

### 2.4 Reactivity of commercially available anti-horse IgG antibodies with the reqIgGs

The following antibodies were tested for reactivity against the reqIgGs in ELISA: goat HRP-conjugated polyclonal antibodies specific for horse IgGa, IgGb, IgGc or IgG(T), (kindly provided by Serotec, Oxford, UK and Bethyl Laboratories, Montgomery, TX, USA), and mouse monoclonal antibodies (mAb) against horse IgGa (CVS48), IgGb (CVS39), IgGc (CVS53) and IgG(T) (CVS38) (kindly provided by Serotec). Secondary antibody used to detect binding of the mAb was a goat anti-mouse IgG1-HRP conjugate diluted 1/10,000 (kindly provided by Serotec). In addition, HRP-conjugated goat polyclonal anti-horse IgG H + L chain (kindly provided by Bethyl Laboratories) and goat anti-horse IgG Fc (Rockland) were tested in ELISA. Antigen-capture ELISAs were performed as above using 250 ng/ml of each purified reqIgG subclass. Detection antibodies were diluted 1/10,000 (goat polyclonals) or 1/100 (anti-IgGa mAb), 1/200 (anti-IgGb mAb), 1/10 (anti-IgGc mAb) and 1/500 (anti-IgG(T) mAb). The goat polyclonal anti-horse IgGa, IgGb, IgGc and IgG(T) antibodies were also tested in immunoblotting. Purified reqIgGs (1 μg) were electrophoresed under reducing and non-reducing conditions and the detection antibodies were diluted as for ELISA.

### 2.5 Analysis of reqIgG glycosylation

ReqIgGs (1 μg) were electrophoresed on 8.4% acrylamide gels under reducing conditions alone or following reduction and de-glycosylation. Removal of *N*-linked sugars was carried out using a GlycoPro enzymatic deglycosylation kit (Prozyme, Inc., Leandro, CA, USA) according to the manufacturer's instructions. Following transfer to nitrocellulose, membranes were probed with the appropriate HRP-conjugated goat anti-horse IgG subclass antibody or either Con A-biotin (diluted 1/10,000) or jacalin-biotin (diluted 1/5000) (both Vector Laboratories, Inc., Burlingame, CA, USA) followed by streptavidin-AP (Dako, Ely, UK). Recombinant human IgG1 and IgA1 (Pleass et al., 1999) were used as positive controls.

### 2.6 Interaction with staphylococcal protein A and streptococcal protein G

Interaction of reqIgGs with protein A and protein G was analysed by ELISA. NIP-BSA coated wells were incubated with 100 μl (0.25 μg/ml) of one of the purified reqIgGs or recombinant human IgG1 for comparison. Binding to protein A or protein G was detected by incubation with 100 μl of serial dilutions of either HRP-conjugated protein A (0–50 μg/ml in PBS-T) or HRP-conjugated protein G (0–5 μg/ml in PBS-T) (both Sigma, Poole, UK). Plates were developed with ABTS and absorbance read at 405 nm.

### 2.7 Functional assays

Chemiluminescence assays were carried out as previously described (Pleass et al., 1999) using 10 μg/ml of each reqIgG and equine PBLs, isolated from blood drawn under appropriate licence from the UK Home Office. Complement binding and activation was assessed by ELISA on NIP-BSA coated wells incubated with recombinant human IgG3 (Bruggemann et al., 1987) or each of the reqIgGs (0–10 μg/ml in PBS-T, 100 μl/well) for 1 h at room temperature. Following washing, plates were incubated with human serum diluted 1/100 in veronal buffered saline containing 0.5 mM MgCl_2_, 2 mM CaCl_2_, 0.05% Tween-20, 0.1% gelatin and 0.5% BSA for 1 h at room temperature. After washing, plates were incubated with either a 1/800 dilution of sheep anti-C1q-HRP (Serotec) or a 1/500 dilution of biotin-conjugated anti-C5b-9 (Quidel, Santa Clara, CA, USA), followed by streptavidin-HRP (Dako) diluted 1/1000 in PBS-T, 0.5% BSA for 1 h at room temperature. Plates were developed as above.

## 3 Results

### 3.1 Analysis of purified antibody by SDS-PAGE and Western blotting

Transfection of each of the equine γ1–γ7 H chain expression vectors into CHO cells stably expressing a compatible mouse λ light (L) chain allowed expression of all seven subclasses. Expressed Ig was purified by antigen affinity chromatography followed by FPLC. All seven IgGs eluted from FPLC as a single major peak representing monomer. Minor peaks eluting earlier were attributed to antibody that had aggregated during purification. For each subclass, fractions corresponding to the major peak were pooled and used for all subsequent experiments.

SDS-PAGE analysis of FPLC purified reqIgGs confirmed that the reqIgs assembled into intact Igs stabilised by interchain disulphide bridges (Fig. 1A). Under reducing conditions, analysis of the seven IgGs revealed that the IgG2 H chain migrated the most quickly, followed closely by those of IgG4 and IgG7, then IgG6, IgG1, IgG5 and IgG3 (Fig. 1B). Under the more sensitive conditions of Western blotting using an anti-mouse λ L chain antibody to detect the horse IgGs (Fig. 1C), some lower molecular weight species were noted for IgG4 and IgG7 under non-reducing conditions. These may represent species such as half molecules (HL) and L chain dimers (L_2_), suggesting that a small proportion of the IgG4 and IgG7 molecules lack inter-H and/or H–L disulphide bonds and are stabilized by non-covalent interactions alone. Hence, under the native conditions of FPLC only a single major peak of fully assembled IgG was seen.

### 3.2 Reactivity of anti-horse IgG antibodies with the reqIgG subclasses

Currently available anti-horse IgG antibodies are categorised on the basis of reactivity against horse IgG subclasses defined under the previous nomenclature of IgGa, IgGb, IgGc, and IgG(T). We sought to analyse the reactivity of these antibodies with the seven reqIgG subclasses. The results, obtained by ELISA, are summarised in Table 1. The polyclonal antibody directed against horse IgGa was specific for a single subclass, namely IgG1. Similarly a polyclonal antibody preparation directed against IgGc was found to recognise just one subclass, in this case IgG6. Goat anti-horse IgGb showed strong reactivity with IgG4 and IgG7 but also weakly recognised IgG1. The goat anti-horse IgG(T) polyclonal antibody reacted most strongly with IgG5, but also recognised IgG2 and IgG3. The pattern of recognition of the IgG subclasses by the mAbs was similar to that of the polyclonal antibodies except that anti-horse IgGb mAb recognised IgG4 and IgG7 but not IgG1, and anti-horse IgG(T) mAb strongly recognised IgG5, weakly recognised IgG3 but showed no reactivity with IgG2. Reactivity of both the polyclonal and monoclonal anti-IgGb antibodies with IgG4 and IgG7 is not surprising as these two subclasses show 97% amino acid identity.

The polyclonal anti-horse IgG (H + L) and anti-horse IgG Fc antibodies recognised all seven IgG subclasses but gave varying signal strengths in the ELISA (see Table 1). Anti-horse IgG (H + L) gave a strong ELISA signal with IgG1, IgG4, IgG5 and IgG7, an intermediate signal with IgG2 and IgG3, and only a weak signal with IgG6. The observed reactivity is directed towards the heavy chain of the recombinant IgGs only, because no binding of the anti-horse IgG (H + L) was seen with recombinant forms of either equine IgA or human IgA (Morton et al., 1993), both of which carry identical light chains to those of the eqIgGs (data not shown). Anti-horse IgG Fc gave strong ELISA signals with IgG1, IgG4 and IgG7, intermediate signals with IgG3 and IgG5, and only weak signals with IgG2 and IgG6.

The reactivities of the anti-horse polyclonal Abs with the horse IgG subclasses when assessed by immunoblotting under non-reducing conditions (Fig. 2A) mirrored those of ELISA. However, under reducing conditions (Fig. 2B) goat anti-horse IgGb recognised IgG4 and 7 but no longer recognised IgG1, suggesting that the IgG1 epitope(s) recognised by this antibody may be discontinuous and depend on the intact disulphide-stabilised structure of the antibody. Several previously described anti-equine IgG monoclonal antibodies were thought to recognise conformational epitopes on equine IgG as they functioned under native conditions but not in immunoblotting (Sheoran et al., 1998). Under reducing conditions, goat anti-horse IgG(T) used at a 1/10,000 dilution recognised IgG3 and 5 but in contrast to non-reducing SDS-PAGE and ELISA no longer reacted with IgG2 but with IgG1 instead. However, recognition of IgG2 under reducing conditions could be achieved with a higher concentration (1/1000 dilution) of detection antibody (data not shown).

Under non-reducing conditions, immunoblotting with goat anti-IgGb (Fig. 2A) revealed additional molecular weight species for IgG4 and IgG7 consistent with those observed with anti-L chain blotting. These additional bands may represent species such as free H-chain, H-chain dimers (H_2_) and half molecules (HL), suggesting, again, an absence of inter-H and/or H–L disulphides in small fractions of these two subclasses.

### 3.3 Analysis of the glycosylation of reqIgGs

All seven reqIgGs contain a conserved potential *N*-glycosylation site within the CH2 domain. Additional potential sites are found in the CH1 domain of IgG3 and IgG5 and in the CH2 domain of IgG2. To determine whether *N*-glycans were attached to any of these sites, the reqIgGs were probed under reducing conditions with concanavalin A (Con A), which is specific for *N*-linked glycans. Con A bound to all reqIgG subclasses confirming that the IgGs are indeed *N*-glycosylated (Fig. 3A). There was, however, some difference in the intensity of the bands, with IgG2 and IgG3 blotting more weakly than the other subclasses, most likely a reflection of the number, type or accessibility of *N*-glycans present.

By contrast, jacalin, which is specific for *O*-linked glycans, bound only to reqIgG3 and to the *O*-glycosylated human IgA1 used as a positive control (Fig. 3B).

Treatment of reqIgGs with *N*-glycanase resulted in a noticeable reduction in the molecular weights of their H chains (Fig. 4), confirming their *N*-glycosylation status. For the IgG2 subclass, reactivity of the detecting antibody (goat anti-horse IgG(T)) was lost following the removal of *N*-glycans, suggesting that the epitopes recognized by this anti-horse reagent are in some way glycan-dependent. The IgG5 H chain migrated as two discrete bands following treatment with *N*-glycanase, possibly reflecting partial removal of the two potential *N*-linked glycans in a proportion of the molecules treated.

### 3.4 Interaction with staphylococcal protein A and streptococcal protein G

Binding of protein A to reqIgGs was generally much weaker than the binding of protein G (Fig. 5), in keeping with earlier reports (Sheoran and Holmes, 1996; Burton and Woof, 1992). A 10-fold higher concentration range of protein A than protein G was required to see significant binding to equine and human IgG.

Protein A showed the highest level of binding to IgG1 and relatively low levels of binding to the other subclasses in the order: IgG3 > IgG4 > IgG7 > IgG5 = IgG2 > IgG6. Sheoran and Holmes (1996) reported moderate adherence of protein A to serum IgGa (i.e., IgG1) but saw no binding of IgGb (IgG4 and 7) or IgG(T) (IgG3 and IgG5). The fact that slight binding of protein A to IgG3, IgG4, IgG5 and IgG7 was observed in our study may be explained by the use of high concentrations of protein A (up to 50 μg/ml) and a sensitive method of assessing the interaction. Sugiura et al. (2000) also reported some binding of equine IgGb and IgG(T) to protein A. In agreement with previous work (Sheoran and Holmes, 1996; Sugiura et al., 2000), binding of IgG6 to protein A was barely detectable above background levels.

Protein G showed strong binding to IgG4 and IgG7, closely followed by IgG1. IgG3 displayed intermediate binding, while binding to IgG6 and IgG2 was low, and IgG5 did not bind. Sheoran and Holmes (1996) also showed that the binding affinity of IgGb (IgG4 and IgG7) to protein G was higher than that of IgGa (IgG1). Furthermore, they identified two fractions of IgG(T), one which bound strongly to protein G and one that bound weakly, which most likely correspond to IgG3 and IgG5, respectively.

### 3.5 Functional assays

We studied FcγR-mediated cellular responses by assessing the capacity of the antibodies to trigger a respiratory burst in equine peripheral blood leukocytes (PBL). Recombinant IgG1, IgG4, IgG5 and IgG7, and to a lesser extent IgG3, all triggered strong respiratory bursts, whereas IgG2 and IgG6 elicited only very weak responses (Fig. 6).

Binding of C1q and activation of the classical complement pathway by the reqIgGs was assessed using ELISA. Human serum was used as a source of complement due to the ready availability of antibodies to detect human C1q and human C5-9 complex. The C1q–IgG interaction is highly conserved throughout evolution and C1q is known to react with IgG from different species (Burton and Woof, 1992). The ability of the reqIgGs to bind C1q (Fig. 7A) was reflected in their ability to activate the classical complement pathway to its terminal components (Fig. 7B). In control experiments, both C1q binding and C5-9 deposition were reduced to zero for all IgGs following heat inactivation of serum (data not shown). IgG3 was the most potent activator of complement, followed by IgG1, IgG4 and IgG7, which all bound C1q and activated complement to the same extent. Recombinant IgG2, IgG5 and IgG6 did not bind C1q or activate complement.

## 4 Discussion

Our studies show that the CHO expression system previously described for human antibodies (Morton et al., 1993) can be used to generate a stable supply of equine IgG antibodies. These recombinant IgGs retain affinity for their antigen, are recognised by anti-mouse λ L-chain and anti-horse IgG antibodies, are glycosylated, and assemble as covalently stabilised four chain (H_2_L_2_) molecules with the expected relative molecular weight of approximately 150 kDa. Hence, in terms of structure, they appear to be representative of natural horse IgGs.

Interestingly, horse IgG3 appears to have *O*-linked as well as *N*-linked glycans attached to the H chain. *O*-glycosylated forms of rabbit IgG and mouse IgG2b in which the *O*-glycans are attached to the hinge region have been described (Fanger and Smyth, 1972a, 1972b; Kim et al., 1994; Kabir et al., 1995). Serine and threonine residues, often in clusters, are known sites for *O*-glycan attachment. A prominent feature of *O*-glycosylation sites is an increased frequency of proline residues, especially at positions −1 or +3 relative to the glycosylated residue (Wilson et al., 1991). The horse IgG3 hinge is rich in proline and threonine and contains two Thr residues with a Pro at position −1 and a number of Thr residues with a Pro at position +3. Hence, it is probable that *O*-glycans are attached to the hinge region of horse IgG3. *O*-glycosylation of the hinge region of IgG confers an increased resistance to proteolysis by various proteases including pepsin, papain and elastase (Fanger and Smyth, 1972b; Kabir et al., 1995; Parham, 1983) and therefore may play a role in protection of eqIgG3 from degradation.

A minor feature of both equine IgG4 and IgG7 was the presence of species such as free H chain, H chain dimers (H_2_), half molecules (HL) and L chain dimers (L_2_) under denaturing conditions, suggesting that a small proportion of the molecules lack H–L or H–H disulphide bonds, akin to human IgA2m(1) and human IgG4, respectively. The human IgG2, IgG3 and IgG4 subclasses are disulphide bonded to the L chain through Cys131 in the CH1 domain. The equivalent Cys is missing in equine IgG4 and IgG7, and may account for the tendency for a minor proportion of these subclasses to exist in forms lacking H–L bonds. The majority of equine IgG4 and IgG7 molecules are present at molecular weights corresponding to intact (H_2_L_2_) antibodies, suggesting that H–L disulphide bonds can exist. Human IgG1, which lacks Cys131 in the CH1 domain, instead forms a disulphide bond to the L chain through Cys220 in the upper hinge (Burton and Woof, 1992). Hence, it is feasible that hinge cysteines in equine IgG4 and IgG7 may participate in H–L disulphide bond formation. Likewise, this could be the case for equine IgG6, which also lacks the corresponding CH1 Cys residue. The appearance of half molecules of equine IgG4 and IgG7 would suggest that a fraction of both these subclasses lack inter-H chain disulphide bonds, with the molecules being stabilised by non-covalent interactions instead. This arrangement has already been noted in a fraction of human IgG4 molecules which are seen as HL half molecules under denaturing, non-reducing conditions (Aalberse and Schuurman, 2002). The deficiency in inter-H-chain bonds in human IgG4 has been attributed to a Ser within the core hinge sequence (CPSC), which replaces the Pro (CPPC) found in isotypes such as human IgG1 and IgG2 that do not have this deficiency. This Ser seems to increase the likelihood that the two core hinge Cys residues form intra- rather than interchain disulphide bonds possibly due to greater hinge flexibility (Angal et al., 1993; Bloom et al., 1997). In equine IgG1, IgG3, IgG5 and IgG6, which all form disulphide bonded H_2_L_2_ molecules, the corresponding core hinge sequence is CPKC. In contrast, the core hinge sequences of eqIgG7 and IgG4 are CPTC and CPAEC respectively, suggesting that deviations from central Lys to either Thr or Ala-Glu may decrease the efficiency of interchain disulphide bridge formation in some way.

Our results for the binding of the reqIgGs to protein A and protein G agree well with those for the binding of horse IgG subclasses which had been purified from serum and classified under the previous nomenclature (Sheoran and Holmes, 1996; Sugiura et al., 2000). The binding sites for protein A and G on the human IgG Fc lie at the CH2-CH3 domain interface, with considerable but incomplete overlap (Deisenhofer, 1981; Sauer-Eriksson et al., 1995) (Fig. 8). The amino acid sequences of equine IgG2, IgG3, IgG4, IgG5, IgG6 and IgG7 all contain at least one amino acid difference from human IgG1 within the regions contributing to protein A binding (Fig. 8). These differences may be sufficient to explain the low affinity of these IgGs for protein A because a single amino acid substitution of His to Arg at position 435 in a human IgG3 allotype is known to prevent binding to protein A (Burton and Woof, 1992). Similarly the differential reactivity of the subclasses with protein G can be rationalized on the basis of amino acid substitutions at key positions in the protein G interaction site (Fig. 8). The fact that the highest level of binding is seen with eqIgG1, IgG4 and IgG7, which like human IgG1 all possess His433 and Tyr436, may suggest that these two residues play key discriminatory roles in the binding of horse IgGs to protein G.

IgGs mediate effector function through interaction with leukocyte FcγRs and activation of the classical pathway of complement. These effector functions differ with IgG subclass (Burton and Woof, 1992). There is little available information with regard to comparative binding of the horse IgG subclasses to FcγRs. An early study found that eqIgG (subclass unspecified) but not eqIgG(T) (i.e., eqIgG3 and/or IgG5) was able to interact via the Fc region with equine monocytes and neutrophils (Banks and McGuire, 1975). In the present study, we have demonstrated that equine IgG1, IgG3, IgG4, IgG5 and IgG7 are able to elicit a strong respiratory burst from equine PBL, predicting that these five subclasses can interact with FcγR on the surface of these cells. IgG2 and IgG6 stimulated little or no response suggesting that these two subclasses are unable to interact efficiently with FcγR. Several amino acids in the lower hinge region of human IgG1 at the *N*-terminus of the CH2 domain (Leu234-Leu235-Gly236-Gly237-Pro238-Ser239) (Fig. 8) play a central role in binding to human FcγR and deviations from this motif help to explain human IgG subclass specificity for FcγR (Burton and Woof, 1992; Woof and Burton, 2004). In the horse IgGs, IgG1 and IgG3, which elicit bursts, retain this motif while IgG2 and IgG6, which do not elicit bursts, display significant differences from the motif (Fig. 8). Thus, amino acid differences in this region may account, at least in part, for the observed differences in ability to trigger a respiratory burst. However, despite IgG4, IgG5 and IgG7 lacking the full motif, these subclasses are still capable of eliciting strong respiratory bursts, suggesting that regions other than the lower hinge region may influence interaction with at least some classes of equine FcγRs.

Activation of the classical complement pathway by IgG may be initiated through the binding of the first complement component C1q, to two or more adjacent IgG molecules. Human IgG subclasses bind C1q in the rank order IgG3 > IgG1 > IgG2 while IgG4 shows no significant binding (Burton and Woof, 1992). Early studies of equine anti-Lac antibodies (Klinman et al., 1966) using guinea pig complement showed that a preparation comprising IgGa and IgGb (i.e., IgG1, IgG4 and IgG7) was able to fix complement whilst IgGc (i.e., IgG6) was not. The current study confirmed and extended these results. We found that eqIgG3 was the most potent activator of complement, followed by eqIgG1, IgG4 and IgG7, while eqIgG2, IgG5 and IgG6 failed to bind C1q or activate complement. While our results were obtained using human serum as a source of complement, and we cannot rule out the possibility of subtle differences of reactivity with horse complement, we feel that our findings provide a good reflection of the likely relative complement-activating capabilities of the different eqIgG subclasses.

The C1q binding site lies within the CH2 domain of IgG, but appears not to be conserved precisely across species. Glu318, Lys320 and Lys322 are necessary for C1q binding by mouse IgG2b, whilst in human IgG1 or IgG3 Asp270, Lys322, Pro329 and Pro331 appear important with minimal contribution from Glu318 and Lys320 (Duncan and Winter, 1988; Idusogie et al., 2000; Thomessen et al., 2000). A comparison of the equine IgG CH2 amino acid sequences does not reveal a common difference between the complement activating and non-activating subclasses at the residues corresponding to Asp270, Glu318, Lys320, Pro329 or Pro331 (Fig. 8). However, all of the complement-activating subclasses have a Lys corresponding to Lys322. The fact that this residue is a serine in eqIgG2 and IgG5 may account, at least in part, for the inability of these subclasses to activate complement. Curiously, IgG6, which possesses a lysine at position 322, does not activate complement, underlining the subtle species differences that are apparent in complement activation.

Our data on the effector function capabilities of the IgG subclasses have important new implications for the design of effective horse vaccines. It is clear that to achieve maximal protection via FcγR- and complement-mediated elimination mechanisms, vaccines should seek to elicit IgG antibodies of the IgG1, IgG3, IgG4 and IgG7 subclasses. Vaccines that trigger only IgG2, IgG5 or IgG6 antibodies are predicted to offer less effective protection. Since IgG plays key roles in both serum and mucosal compartments in the horse, these considerations are applicable to both systemic and mucosal vaccination strategies.

Further, our findings on the relative effector function capabilities of the different IgG subclasses lend themselves to a rationalization of the protection offered by natural IgG immune responses against various infectious agents. Thus, investigations into the role of individual subclasses in protective immunity have demonstrated that IgGa and IgGb (i.e., the FcγR- and complement-engaging isotypes IgG1, IgG4 and IgG7) contribute to protection against equine influenza virus (Nelson et al., 1998; Breathnach et al., 2006; Soboll et al., 2003), *Streptococcus equi* (Sheoran et al., 1997) and *Rhodococcus equi* (Lopez et al., 2002). Indeed, IgGb (IgG4 and IgG7) has been suggested to be most important in equine protective antibody-mediated immune responses to intracellular pathogens (Nelson et al., 1998; Lopez et al., 2002; Goodman et al., 2006), whereas IgGc (IgG6) is suggested to be least important (Sheoran et al., 2000). The current study helps rationalize this observation as both IgG4 and IgG7 are able to stimulate a potent respiratory burst and activate complement via the classical pathway. By contrast, these effector functions are absent in the IgGc (IgG6) subclass. The requirement of equine IgGs to recruit effector molecules for effective immunity is illustrated by several studies. For example, IgG-mediated neutralisation of equine arteritis virus (EAV) (Balasuriya and MacLachlan, 2004) and acute phase EHV-1 (Snyder et al., 1981) is complement dependent, and opsonisation by specific IgG is necessary for efficient phagocytosis of *Rhodococcus equi*, *Escherichia coli* and *Actinobacillus equuli* by equine neutrophils or alveolar macrophages (Hietala and Ardans, 1987; Grondahl et al., 2001; Cauchard et al., 2004). Drawing all this information together, it is clear that the enhanced effector function capabilities of equine IgG1, IgG3, IgG4 and IgG7 equip these subclasses for key protective roles.

International meetings have highlighted the need for further research into the functional roles of equine IgG subclasses and for the development of tools to study equine Igs (Lunn et al., 1998). The reqIgGs described here are a reliable source of pure and homogeneous equine IgG subclasses and will serve as useful reference proteins for the production and screening of equine specific reagents. In particular, the generation of mAb able to discriminate between the seven subclasses is an ongoing project. Moreover, they will provide a valuable resource for future research, in particular in delineation of the function of individual IgG subclasses in antibody-mediated immunity of the horse.

## Figures and Tables

**Fig. 1:** SDS-PAGE analysis of purified reqIgGs. ReqIgGs were analysed by SDS-PAGE and stained with Coomassie under (A) non-reducing conditions and (B) reducing conditions. (C) Immunoblot analysis under non-reducing conditions probed with rabbit anti-mouse λ L chain cross out (C). sIgG, horse serum IgG; huIgG, recombinant human IgG1 containing mouse λ L chains. On each gel, an equivalent quantity of each reqIgG subclass was loaded (5 μg for Coomassie stained gels and 1 μg for immunoblots). The “doublet” bands apparent in some subclasses under non-reducing conditions probably reflect heterogeneity in glycosylation.

**Fig. 2:** Reactivity of polyclonal anti-horse IgG subclass antibodies with reqIgGs in immunoblotting under (A) non-reducing conditions and (B) reducing conditions. Numbers at the top refer to the subclass loaded in that lane. The anti-IgG subclass antibody used is indicated below each image. On each gel, an equivalent quantity of each reqIgG subclass (1 μg) was loaded.

**Fig. 3:** Reactivity of reqIgGs with Con A (A) and jacalin (B). huIgG1, recombinant human IgG1; huIgA1, recombinant human IgA1. On each gel, an equivalent quantity of each reqIgG subclass (1 μg) was loaded.

**Fig. 4:** Immunoblot of reqIgGs under reducing conditions untreated or treated with *N*-glycanase. C, control untreated IgG; T, treated with *N*-glycanase. IgG1 was probed with anti-horse IgGa; IgG2, IgG3 and IgG5 with anti-horse IgG(T); IgG4 and IgG7 with anti-horse IgGb; and IgG6 with anti-horse IgGc. On each gel, an equivalent quantity of each reqIgG subclass (1 μg) was loaded.

**Fig. 5:** ELISA analysis of protein A (A) and protein G (B) binding to equivalent quantities of the reqIgG subclasses. The means of three experiments are shown. Standard error was <5% between experiments. huIgG1, recombinant human IgG1.

**Fig. 6:** Stimulation of respiratory burst in equine PBL by equivalent quantities of the reqIgG subclasses. Each point is the mean of triplicate determinations. The experiment was performed three times with PBL from different donors. The results shown are those from a typical experiment. RLU, relative light index.

**Fig. 7:** C1q binding (A) and C5-9 deposition (B) by antigen-captured reqIgG as detected by ELISA. huIgG3, recombinant human IgG3. The figure shows the mean of three experiments.

**Fig. 8:** Amino acid sequence alignment of the Fc region of eqIgGs. The sequence of human IgG1 Fc is shown for comparison. Human IgG1 residues implicated in interactions are indicated as follows: protein A, bold, italic; protein G, bold, non-italic; both protein A and protein G, box; FcγR, grey highlight; C1q, underline.

**Table 1:** Reactivity of anti-horse IgG antibodies with reqIgGs

	IgG1	IgG2	IgG3	IgG4	IgG5	IgG6	IgG7
Goat polyclonal							
anti-IgGa	+++						
anti-IgGb	+			+++			+++
anti-IgGc						+++	
anti-IgG(T)		++	+		+++		

Mouse monoclonal							
anti-IgGa (CVS48)	+++						
anti-IgGb (CVS39)				+++			+++
anti-IgGc (CVS53)						+++	
anti-IgG(T) (CVS38)			+		+++		

Goat anti-horse IgG (H + L) (Bethyl)	+++	++	++	+++	+++	+	+++

Goat anti-horse IgG Fc (Rockland)	+++	+	++	+++	++	+	+++

+++ Strong reactivity.

++ Intermediate reactivity.

+ Weak reactivity.
